# The Compound Effect of Spatial and Temporal Resolutions on the Accuracy of Urban Flood Simulation

**DOI:** 10.1155/2022/3436634

**Published:** 2022-06-08

**Authors:** Xiting Li, Leizhi Wang, Haolan Zhou, Yintang Wang, Kaijie Niu, Lingjie Li

**Affiliations:** ^1^Tianjin University, Tianjin 300350, China; ^2^Nanjing Hydraulic Research Institute, Nanjing, Jiangsu 210029, China; ^3^South China Agricultural University, Guangzhou, Guangdong 510642, China

## Abstract

Flood disaster is one of the critical threats to cities. With the intellectualization tendency of Industry 4.0, refined urban flood models can effectively reproduce flood inundation scenarios and support the decision-making on the response to the flood. However, the spatiotemporal variability of rainfall and the spatial heterogeneity of the surface greatly increase the uncertainties in urban flood simulations. Therefore, it is crucial to account for spatiotemporal variability of rainfall events and grids of the model as accurately as possible to avoid misleading simulation results. This study aims to investigate the effect of temporal resolutions of rainfall and spatial resolutions of the model on urban flood modeling in small urban catchments and to explore a proper combination of spatiotemporal schemes. The IFMS Urban (integrated flood modeling system, urban) is used to construct a one-dimension and two-dimension coupled urban flood model in the typical inundated area in Dongguan, China. Based on five temporal resolutions of rainfall input and four spatial resolutions, the compound effect of spatiotemporal resolutions on the accuracy of urban flood simulations is systematically analyzed, and the variation characteristics are investigated. The results show that the finer the temporal resolution is, the higher the simulation accuracy of the maximum inundated water depth. Considering the spatial resolution, as the spatial grid becomes smaller, the relative error of the maximum inundated water depth decreases, but it also shows some nonlinear characteristics. Therefore, the smaller grid does not always mean a better simulation. The spatial resolution has a greater impact on the flood simulation accuracy than the temporal resolution. The simulation performance reaches the best when the grid interval is 100 m and the rainfall input interval is 5 min, 10 min, or 15 min. Affected by other factors such as terrain slope, the simulation accuracies under different spatiotemporal resolutions present complex nonlinear characteristics. The mechanisms of the compound effect of the spatiotemporal resolutions on the model simulation and the effect of underlying surface and topography on model simulation will be the focus of in-depth exploration for the future urban flood model.

## 1. Introduction

With booming urbanization, the flood-inducing factors and hazard bearing bodies have experienced great changes in recent years. Many large and medium-sized cities around the world have suffered from frequent floods, which seriously threaten the safety of life and property of urban residents [1–3]. As an important basis for urban flood emergency control and risk management, the urban flood model is very important in real-time simulation, early warning, and risk assessment of floods. In recent years, under the background of Industry 4.0, the algorithms, calculation data, and computing power have greatly improved [4]. The spatiotemporal resolutions of urban flood models are becoming higher, and the decision-making is more intelligent. However, the fine-resolution simulation brings computational pressure and increases the uncertainties in the urban flood simulation. Due to the diverse underlying urban surface, the fast runoff process, and the short response time, its hydrological characteristics in urban regions show high spatiotemporal heterogeneity [5, 6]. Therefore, the urban flood model generally has strong resolution dependence, and the simulation accuracy is constrained by the spatiotemporal resolutions [7–9]. To improve the simulation accuracy, we need to conduct in-depth and systematic research on the impact of spatiotemporal resolutions on the simulation accuracy of urban flood models.

Rainfall is one of the key driving factors of urban hydrological processes and is of high spatiotemporal variability [10, 11]. Variations of the rainfall spatiotemporal resolutions can affect the rainfall-runoff response time and water yield in the hydrological model [11]. Therefore, it is important to simulate the hydrological response with an appropriate spatiotemporal resolution of rainfall [12, 13]. A large number of studies have proved that for small urban catchments, urban flood simulation should use the rainfall data on at least 1–15 min time resolution and 100–1000 m spatial resolution [14–16]. Bruni et al. [17] analyzed the relationship between the urban catchment area and the required spatiotemporal resolutions of rainfall data and showed that for small urban catchments with less than 700 hectares, the urban hydrological simulation requires the rainfall data with at least a 5 min time resolution and a 1.7 km spatial resolution. In addition, the sensitivity of different hydrological models to the spatiotemporal resolutions of rainfall differs significantly, with the physical model being more sensitive than the conceptual model [18–20]. Aronica et al. [21] found that the Storm Water Management Model (SWMM) is more sensitive to rainfall temporal resolution than hydrological parameters. Meselhe et al. [22] compared the HMS (hydrologic modeling system) conceptual model with the physics-based hydrological model MIKE SHE. They found that the latter is more sensitive to rainfall temporal resolution. Gires et al. [23] found that the 1D/2D (one-dimension/two-dimension) coupled model, Multi-Hydro, is more sensitive to rainfall variability than the simpler 1D model. Many other studies also found that in small urban catchments, the time-scale variation of rainfall data has a greater impact on urban hydrodynamic models [24, 25]. To sum up, for a densely built and highly impermeable urban catchment, the output of the urban flood model is very sensitive to the rainfall spatiotemporal resolutions, and the bias of output increases obviously as the resolutions decrease.

Most urban flood models are distributed hydrological models based on grid data. The hydrological process is also sensitive to the spatial distribution of the underlying surface of the watershed [9]. The computational efficiency of the model and the accuracy of the simulations are often affected by the spatial resolution of the grid and the accuracy of input data [26, 27]. In the early 1960s, the importance of the spatial resolution of input data is recognized by scholars [28, 29]. Since then, many scholars have studied the spatial resolution of hydrological models. They found that the conclusions are different in different study areas. The model of high spatial resolution can lead to the systematic underestimation of peak flow [30, 31]. Ichiba et al. [27] found that increasing spatial resolution can reduce peak flow and total flow. The effect of spatial resolution of the grid on model performance is nonlinear, and higher mesh accuracy does not necessarily lead to better simulation. Zhang and Montgomery [32] found that a spatial resolution of 10 m can greatly improve the simulations than 30 m and 90 m, while that of 2 m or 4 m only improves the model slightly. The above studies show that the difference in spatial resolutions will change the loss of underlying surface information and the complexity of the surface runoff between adjacent grids, which has a nonlinear impact on the simulations. Therefore, in the modeling process of the urban flood, the appropriate spatial resolution should be selected according to the comprehensive analysis of the calculation characteristics of the model, the characteristics of the underlying surface of the study area, and the accuracy of the input data.

To sum up, there have been extensive studies on evaluating the accuracy of urban flood simulation unilaterally from the temporal resolution of rainfall data or spatial resolution of the grids. These studies show that the effects of temporal resolution and spatial resolution on the simulation accuracy are obvious and nonlinear. So, the compound effects of grid spatial resolution and rainfall temporal resolution on the simulation accuracy should be more complicated. However, there are few studies on this aspect. To this end, we take the typical flooded area in Dongguan, China, as the study area (Section 2.1) and collect topographic and sewer network data (Section 2.2). The distributed urban flood model IFMS Urban (Section 3.1) is used to construct the coupling model of the 1D urban drainage network model and 2D surface hydrodynamic model in the study area, and the model is validated by using the high temporal resolution rainfall data and observed historical inundation events (Sections 2.2 and 3.3). Then, we explore the effects of rainfall temporal resolution and model spatial resolution on the maximum inundation water depth and the submerged water depth hydrograph based on five temporal resolutions of rainfall input and four spatial resolutions(Sections 4.1 and 4.2). Furthermore, we analyze the compound effects of different spatiotemporal resolutions on the accuracy of urban flood simulations (Section 4.3). Conclusions can be found in Section 5.

## 2. Study Domain and Data

### 2.1. Study Domain

The study site, Guancheng District of Dongguan City, is located on the south-central east coast of the Pearl River estuary, Guangdong Province, China (within E119°31′-114°15′, N22°39′-23°09′). It covers approximately 13.31 km^2^ (Figure 1(a)). The study area represents a typical urban area with a density of human structures such as houses, commercial buildings, and roads. When the city is hit by heavy rainfall, the topographic characteristics of the study area make the flood converge to the middle from the sides south and north and finally discharge into the Dongyin Canal in the east.

### 2.2. Data Collection

#### 2.2.1. Topographic Data

The basic geographic data provided by the Urban Planning Bureau of Dongguan City (UPBDC) included a remote-sensing image and a digital elevation model (DEM). The resolution of the remote-sensing and DEM are 5 m and 0.5 m, respectively. The former was used to distinguish the land use types of the underlying surface, and the latter was used to calculate the elevation and slope of the 2D grid.

#### 2.2.2. Sewer Network Data

The sewer network data (Figures 1(b) and 1(c)) that were obtained from UPBDC is mainly based on the combined system. Most of the pipelines do not meet the design return period of one year, and most of the pipelines are less than 1000 mm in diameter, which is easy to cause waterlogging in the lower terrain.

#### 2.2.3. Rainfall Data

In this research, two rainstorm events that occurred on August 30, 2018, and May 7, 2015, were used for model calibration and impact study of temporal and spatial scale, respectively. The maximum 24-hour cumulative rainfall of the two rainstorm events exceeded 50 mm, resulting in waterlogging in the study area. Three rainfall stations, which collect rainfall data at an interval of every 5 min, are located in and around the study area (Figure 1(c)). The rainfall of 10 min, 15 min, 30 min, and 1 h temporal scale was accumulated from the rainstorm of May 7, 2015. Meteorological Bureau of Dongguan City provided the corresponding rainfall records.

#### 2.2.4. Observed Historical Inundation Events

Generally, it is difficult to calibrate and validate the urban inundation model due to a lack of detailed observation of inundation events [2]. Therefore, in many cases, either a partial calibration/validation of the model or an indirect validation/verification based on testimonial reports is sought [33, 34]. In this research, the process of inundation depth in the inundation area in Yonghuating, Dongcheng Road West, and Dongzong Road on August 30, 2018, was observed for the calibration and verification of the urban flood model. The data on maximum inundation depth and distribution of inundation area on May 7, 2015, were collected and released by the Water Authority of Dongguan City.

## 3. Methodology

### 3.1. IFMS Urban

IFMS Urban couples the SWMM with a 2D surface hydrodynamic model that is conducted based on an adaptive grid and finite volume method, which can automatically identify the region with a large parameter gradient and the boundary between dry and wet, adjust the grid size, accurately simulate the dynamic change of water flow propagation, and can be applied to the actual flood simulation [35]. The IFMS Urban efficiently calculates the urban flood process in the complex urban area with frequent waterlogging and achieves good calculation accuracy, which provides technical support for this paper.

#### 3.1.1. 1D Urban Drainage Network Model

The urban drainage system consists of water inlets, drainage pipes, drainage pumping stations, and river channels at the outlets of the pipe network. The 1D model can use three methods of dynamic wave method, kinematic wave method, and steady flow method to calculate the drainage pipeline confluence. The governing equation is specifically the following formulas:

(1) $$\begin{array}{c} \frac{\partial Q}{\partial x}+\frac{\partial A}{\partial t}=0, \end{array}$$

where *Q* is the discharge, *A* is the discharge section area, *t* represents the time, and *x* represents the distance.

(2) $$\begin{array}{c} gA\frac{\partial H}{\partial x}+\frac{\partial \left(Q^{2}/A\right)}{\partial x}+\frac{\partial Q}{\partial t}+gAS_{f}=0, \end{array}$$

where *H* represents the water depth, *g* represents the gravitational acceleration, and *S*_*f*_ is the slope gradient of friction resistance.

#### 3.1.2. 2D Surface Hydrodynamic Model

In order to establish a special well-balanced scheme technique for dealing with source term due to bottom topography constructed, this paper develops a well-balanced Godunov-type scheme of the second-order accuracy for 2D shallow water equation with mesh. As above, the MUSCL method is used to reconstruct the variable values on both sides of the unit interface *U*_*i*+1/2_^*L*/*R*^ and the Roe format is selected to solve interface flux in the evolutionary step. Regarding the discretization of the source term, the bed slope term is discretized by characteristic classification, and the resistance source term is discretized implicitly.

The 2D shallow water equation of depth-averaged can be abbreviated as follows:

(3) $$\begin{array}{c} \frac{\partial h}{\partial t}+\frac{\partial hu}{\partial x}+\frac{\partial hv}{\partial y}=0,\\ \frac{\partial hu}{\partial t}+\frac{\partial }{\partial x}\left[hu^{2}+\frac{1}{2}gh^{2}\right]+\frac{\partial huv}{\partial y}=S_{x},\\ \frac{\partial hu}{\partial t}+\frac{\partial hvu}{\partial x}+\frac{\partial }{\partial y}\left[hv^{2}+\frac{1}{2}gh^{2}\right]=S_{y}, \end{array}$$

where *h* represents the water depth, *u* is the flow velocity of *x*-direction, *v* is the flow velocity of *y*-direction; *S*_*x*_ and *S*_*y*_ are the source terms.

#### 3.1.3. Algorithm of Coupled Model

The 1D urban drainage network model and 2D surface hydrodynamic model are coupled by calculating the exchange water volume, which is substituted into their respective model for calculation and update to the next step. The exchange water volume can be calculated through the following equation:

(4) $$\begin{array}{c} Q=M\left(H_{\text{node}}-H_{\text{surface}}\right)W_{\text{crest}}\sqrt{2g\left|H_{\text{node}}-H_{\text{surface}}\right|}\frac{\left|H_{\text{node}}-H_{\text{surface}}\right|}{\left|\max\left(H_{\text{node}},H_{\text{surface}}\right)-H_{g}\right|}, \end{array}$$

where *H*_Surface_ is the head of land surface, *H*_node_ is the head of drainage pipeline, *M* is the discharge coefficient, *W*_crest_ is the width or perimeter of manhole, and *H*_*g*_ is the surface elevation.

### 3.2. Evaluation of Modeling Results

The calibration process has been evaluated using error indicators including Nash-Sutcliffe efficiency coefficient (NSE), maximum inundation depth relative error (RE_*P*_) , and maximum inundation depth appearance time absolute error (AE_*T*_) for the simulated and observed values. The error indicators are formulated as in the following equations:

(5) $$\begin{array}{c} \text{NSE}=1-\frac{\sum_{i=1}^{N}{\left(q_{i}^{\text{obs}}-q_{i}^{\text{sim}}\right)}^{2}}{\sum_{i=1}^{N}{\left(q_{i}^{\text{obs}}-{\bar{q}}^{\text{obs}}\right)}^{2}}, \end{array}$$

where *q*_*i*_^obs^ is the observed value of an event *i*, *q*_*i*_^sim^ is the simulated value of an event *i*, *N* is the number of observed values, and ${\bar{q}}^{\text{obs}}$ is the average of observed values.

(6) $$\begin{array}{c} {\text{RE}}_{P}=\frac{\left|q_{P}^{\text{obs}}-q_{i}^{\text{sim}}\right|}{q_{P}^{\text{obs}}}\times 100\%, \end{array}$$

where *q*_*P*_^obs^ is the observed value of maximum inundation depth, *q*_*P*_^sim^ is the simulated value of flood peak maximum inundation depth.

(7) $$\begin{array}{c} {\text{AE}}_{T}=T_{P}^{\text{obs}}-T_{P}^{\text{sim}}, \end{array}$$

where *T*_*P*_^obs^ is the observed value of maximum inundation depth appearance time, and *T*_*P*_^sim^ is the simulated value of maximum inundation depth appearance time.

In order to compare the results from different rainfall temporal resolution and 2D grid scale and also to compare the effect of the composition of the rainfall temporal resolution and 2D grid scale, different measures were used. In addition to the common error indicators such as RE_*P*_ and AE_*T*_, we also used the coefficient of determination (*R*^2^) to compare the correlation of two inundation depth series. The closer *R*^2^ to 1, the higher the correlation between the two inundation depth series. *R*^2^ is specifically as follows:

(8) $$\begin{array}{c} R^{2}=\frac{\sum {\left(Y_{A}-\bar{Y_{A}}\right)}^{2}-\sum {\left(Y_{A}-Y_{B}\right)}^{2}}{\sum {\left(Y_{A}-\bar{Y_{A}}\right)}^{2}}, \end{array}$$

where *Y*_*A*_ is the value of the inundation depth series *A*, $\bar{Y_{A}}$ is the mean value of the inundation depth series *A*, and *Y*_*B*_ is the value of the inundation depth series *B*.

### 3.3. Model Validation

#### 3.3.1. Model Setup

The model is set up based on the drainage network. The study area is generalized into 999 pipes, 1011 manholes, and 12 outlets. The parameters for the model include the section size of the drainage network, the two-dimensional (2D) grid elevation, the subcatchment slope, and the 2D grid pervious surface ratio. The section parameters of the drainage network are obtained from the actual survey data. The 2D grid elevation and the subcatchment slope are determined based on the DEM data. The 2D grid pervious surface ratio is extracted from the remote sensing images over the study area. The empirical parameters of the model include the impervious area Manning's roughness, the depression storage for the pervious area, and the infiltration related parameters. The empirical parameters are calibrated according to the SWMM user manual and the hydrogeological characteristics of the study area, as shown in Table 1. The rainwater in the study area flows through the pipeline by gravity and is finally discharged into the Dongyin Canal. According to historical data, the water level of the Dongying Canal is low and does not affect the outflow of the pipeline. Therefore, the model boundary outflow condition is set to free outflow. The modeling time step is set to 20 s, and the total simulation time is 24 h. The setting can ensure that the pipeline network system has no inflow. The accumulated water in the pipeline has been emptied when the simulation ends under each input rainfall condition.

#### 3.3.2. Model Validation

In this section, we validate the IFMS Urban model by using the rain and flood event on August 30, 2018, as an example. The rainfall poured heavily in the study area from 11:00 to 16:00, within which rainfall amount accounted for over 80% of the total in the day. Thus, a 5 h storm event spanning from 11:00 to 16:00 was used as model rainfall data.

A summary of the simulations performed is given in Figure 2 and Table 2. The model can well predict the flood occurring and receding at the typical waterlogging points of Yonghuating, Dongcheng West Road, and Dongzong Road. These results confirm that the simulation of flood processes is reasonably well, with NSE for all waterlogging points exceeding 0.75. The RE_*P*_ and AE_*T*_ ranged approximately from 11.11% to 17.50% and from 5 min to 12 min, respectively. All of them are within the allowable error range required by the Standard for Hydrological Information and Hydrological Forecasting of China. Furthermore, the results of Dongcheng West Road are better than other waterlogging points, with NSE, RE_*P*_ and AE_*T*_ being 0.86, 11.11%, and 5 min, respectively. In conclusion, the above results show that the parameters of the model are set reasonably, and the model has good applicability in the study area. The model is reliable and is suitable for the subsequent analysis.

## 4. Results and Discussion

### 4.1. Effect of Rainfall Temporal Resolution

Table 3 and Figure 3 show the maximum inundation water depth and RE_*P*_ at five typical waterlogging points under five temporal resolutions. With the increase of rainfall temporal resolution, the maximum inundation water depth gradually decreases and RE_*P*_ increases. However, the effect of the rainfall temporal resolution on the maximum inundation water depth is small on the whole. Increasing the time step of rainfall input from 5 min to 30 min, the variation range of the maximum inundation water depth at the five waterlogging points is within 5 cm, while the variation range of RE_*P*_ is less than 8%. RE_*P*_ at waterlogging points based on the 1 h temporal resolution is larger than the other four temporal resolutions, with that in Dongcheng West Road being the largest (13.73%). The errors of the maximum inundation water depth at the waterlogging points increase with the temporal interval of rainfall input, but the overall increase is not large.

The occurrence time of the maximum inundation water depth (referred to as the peak time of inundation water depth) at waterlogging points has a high correlation with the temporal resolution of rainfall input. As shown in Table 4, with the increase of the temporal resolution of rainfall input, the time between the peak time of inundation water depth at waterlogging points and the rainfall peak time (referred to as the lag time) also increases. The lag time of the 10 min and 15 min rainfall input intervals at the five waterlogging points is short (only 0–3 min). The lag time of the 30 min and 1 h rainfall input intervals changes a lot. Compared with the 5 min time interval, the lag time is, respectively, extended by 7–13 min and 23–36 min.

With the increase of rainfall input interval, the correlation between the submerged water depth and the rainfall at waterlogging points decreases. The deformation degree of the submerged water depth hydrograph at waterlogging points becomes larger. Taking the waterlogging point, Yonghuating, as an example (as shown in Figure 4), the rainfall peaks twice at about 1 h and 2 h. Correspondingly, there are two obvious waterlogging processes in 1-2 h and 3-4 h under the 5 min, 10 min, 15 min, and 30 min rainfall temporal resolutions at Yonghuating, and the results have a good correlation with the rainfall observation. The submerged water depth hydrograph under the 1 h rainfall temporal resolution has only one obvious waterlogging process. Compared with the waterlogging processes under other temporal resolutions, the maximum inundation depth is lower and the corresponding occurrence time is later. Using the coefficient of determination (*R*^2^), this study further analyzes how well the shape of submerged water depth hydrographs under 10 min, 15 min, 30 min, and 1 h rainfall input resolutions at five typical waterlogging points match that of the hydrograph under the 5 min resolution (Figure 5). With the increase of temporal interval, the coefficient of determination decreases, and the difference between submerged water depth hydrographs increases. The shape for the 10 min and 15 min resolutions is in good agreement with the submerged water depth process under 5 min resolution, and *R*^2^ are all higher than or equal to 0.97. However, there are certain differences of hydrographs between 1 h and 5 min resolutions, and the *R*^2^ is only 0.69–0.81.

### 4.2. Effect of the 2D Spatial Resolution of Model Grids

The study area is used as the meshing area to generate four kinds of mixed 2D meshes of triangles and quadrilaterals with spatial scales of 50 m × 50 m, 100 m × 100 m, 150 m × 150 m and 200 m × 200 m. According to the remote sensing images, we analyze the land use type of the underlying surface and set the impervious area and roughness of the simulations under four spatial resolutions. The grid elevations for the four spatial resolutions are all obtained by inverse distance weighted interpolation based on a DEM with a resolution of 5 m.

As shown in Table 5 and Figure 6, the effect of grid spatial resolution on the model simulation is nonlinear. It means that the smaller spatial resolution does not correspond to the higher accuracy of model outputs. With the increase of grid spatial interval, the maximum inundation depth decreases and the absolute error (AE) of the maximum inundation depth increases on the whole. When the grid spatial resolution is increased from 50 m to 150 m, the maximum inundation depth decreases, and its variation range is small. All AE is within 4 cm and RE_*P*_ is less than or equal to 6%, while those of the 200 m grid are larger than the other resolution simulations. The maximum inundation depths with a spatial resolution of 50 m at the five typical waterlogging points are all overestimated. Except for Yinshan Street, RE_*P*_ of the 50 m grid is higher than that of the 100 m grid at other four waterlogging points.

There are significant correlations between the slope and the grid spatial resolution of the catchments of waterlogging points and the hydrological characteristics. As the spatial resolution becomes larger, the calculation accuracy of the waterlogging point with large slope of catchment area decreases obviously. The DEM and flow direction of main roads in the study area and around each waterlogging point are shown in Figure 7. On one hand, the three areas of Yinshan Street, Dongzong Road, and People's Park are located in the low-lying central of the study area, where the rain and floods in the eastern, northern, and southern parts of the study area are concentrated. But due to the flat terrain from the Yinshan Street to the People's Park, the converged rain and floodwater cannot be discharged in time, resulting in waterlogging in the three areas. When the grid resolution is increased from 50 m to 200 m, the simulation results at Yinshan Street, Dongzong Road, and People's Park are less affected by the grid size. All AE is less than 3 cm and RE_*P*_ is less than 13%. On the other hand, small-scale rain and floods are gathering in the mountainous southeast of the study area, mainly located in Yonghuating and Dongcheng West Road. The slope in the catchment areas is larger than that in other waterlogging areas. When the grid resolution is increased from 50 m to 150 m, AE and RE_*P*_ in Yonghuating and Dongcheng West Road have a small variation range, while AE and RE_*P*_ at the 200 m grid have increased obviously, reaching 7.07–27.26 cm and 23.6–45.43%, respectively. In the urban flood model, the spatial grid is the basic unit of the runoff calculation of the model. The slope and other properties of the underlying surface have a direct impact on the runoff calculation. In this study, most of the study area is continuous urban hard ground or green space. With the increase of the spatial grid interval, the generalization of the terrain and underlying surface information is greater, and variation details of the urban terrain and underlying surface are covered up. Therefore, the simulations at Yonghuating and Dongcheng West Road where there is larger slope are more affected by the spatial resolution.

### 4.3. The Compound Effect of Rainfall Temporal Resolution and Grid Spatial Resolution

In this study, four rainfall temporal resolutions of 5 min, 10 min, 15 min, and 30 min are selected to be matched with three grid spatial resolutions of 50 m × 50 m, 100 m × 100 m and 150 m × 150 m. Thus, 12 experiments with different spatial and temporal resolutions are conducted. The IFMS Urban model is used to simulate the 12 experiments, and the compound effects of spatiotemporal resolutions on flood simulations have been compared and analyzed.

As shown in Figure 8, the effect of spatial resolution at typical waterlogging points is greater than that of rainfall temporal resolution. For the grids with different resolutions, with the increase of rainfall temporal resolution from 5 min to 30 min, the maximum inundation depth at typical waterlogging points has a small variation range, and RE_*P*_ is less than 3%. The effects of the 5 min, 10 min, and 15 min temporal resolutions are very close. For different rainfall temporal resolutions, with the increase of grid spatial interval, RE_*P*_ at typical waterlogging points greatly changes with nonlinear characteristics. For the waterlogging points of Dongcheng West Road and Yonghuating with a large slope, large grids have a larger influence on the simulation results, while for the flat Dongzong Road and People's Park, small grids have a larger influence on the simulation results.

In urban flood simulation, the finer spatiotemporal resolution does not mean more accurate simulation results. For the 50 m grids, the maximum inundation depth is overestimated under different rainfall temporal resolutions. The finer the temporal resolution is, the greater the overestimation is. At the five typical waterlogging points, RE_*P*_ with the spatiotemporal resolutions of 5 min and 50 m is relatively large, ranging from 1.8% to 10%. In contrast, the water depth range that decreases with the increase of rainfall temporal resolution is small. It is not enough to compensate for the overestimated water depth range under the high-precision grid and RE_*P*_ is still larger than that of the 100 m grid. For the grid of 100 m, the overall simulations are better than those of 50 m and 150 m. The 5 min × 100 m, 10 min × 100 m, and 15 min × 100 m resolutions can achieve the best simulations at different typical waterlogging points, and their RE_*P*_ ranges from 0.3% to 6.1%. For the grid of 150 m, the maximum inundation depth of typical waterlogging points is underestimated. With the increase of rainfall temporal resolution, the maximum inundation depth decreases and the RE_*P*_ increases. By judging the compound effect of rainfall temporal resolution and grid spatial resolution on the simulations, we find the simulation results are better with the 5 min, 10 min, or 15 min rainfall temporal resolution and the 100 m grid spatial resolution.

## 5. Conclusions

This study utilized the IFMS Urban model that couples SWMM and 2D hydrodynamic model to analyze the response of the flood process of urban to different spatiotemporal resolutions. The typical waterlogged area, Guancheng District of Dongguan City, China, was selected as the study area. The variation characteristics of maximum inundation water depth and inundation process were investigated based on five rainfall temporal resolutions and four grid spatial resolutions. The main conclusions are as follows:

With the increase of rainfall temporal resolution, the accuracy of the simulated maximum inundation depth decreases, the time interval between the occurrence of the maximum inundation depth and the peak time of rainfall is prolonged, and the shape of the submerged water depth hydrograph changes greatly, which means the inundation process correlation with the rainfall process is decreased. Compared with the temporal resolution of 5 min, 10 min, 15 min, or 30 min, the 1 h temporal resolution has a greater influence on urban flood simulation.

For the effect of grid spatial resolution, the effect of grid resolution on urban flood simulation is nonlinear. With the increase of grid interval, the maximum inundation depth decreases and RE_*P*_ presents an overall increasing trend. For the fine 2D grids, the maximum inundation depth is overestimated, and the simulations at the waterlogging points with larger slopes are more affected by the spatial resolution.

In this study, the grid spatial resolution has a greater effect on the simulations at typical waterlogging points than the rainfall temporal resolution. It is not the case that the finer spatial and temporal resolutions are, the higher the accuracy of the simulation will be. The simulations perform better with the 5 min, 10 min, or 15 min rainfall temporal resolution and 100 m grid spatial resolution. For the area with the large slope in the catchment areas, using a 2D grid with a smaller grid spatial interval can obviously improve the computational accuracy of the model.

In this study, we have not considered the influence of terrain slope and vertical structure on the urban flood model. In the future, we will focus on the mechanisms of the compound effect of the spatiotemporal resolutions, and on how the model accuracy is affected by the type and slope of underlying surface.

## Figures and Tables

**Figure 1:** (a) Location and landcover conditions of the study area in which five numbers from #1 to #5 labeled with distribution of waterlogging points: #1 People's Park; #2 Dongzong Road; #3 Yinshan Street; #4 Dongcheng West Road; #5 Yonghuating. (b) shows the sewer network with manholes and outlets. (c) Top view of the DEM overlaid with the pipeline and rainfall station layer of the study area.

**Figure 2:** Simulation results of flood processes at typical waterlogging points.

**Figure 3:** Relative errors of maximum inundation water depth (RE_*P*_) at five typical waterlogging points under five rainfall temporal resolutions.

**Figure 4:** The hydrographs of inundation under five rainfall temporal resolutions at Yonghuating.

**Figure 5:** The coefficients of determination of inundation hydrograph between four rainfall temporal resolutions and the 5 min resolution.

**Figure 6:** Variations of RE_*P*_ at typical waterlogging points under four grid spatial resolutions.

**Figure 7:** Topography and flow direction of main roads in the study area (The five waterlogging points numbered #1 to #5 are People's Park, Dongzong Road, Yinshan Street, Dongcheng West Road, and Yonghuating).

**Figure 8:** Bubble charts of the relative error of maximum inundation depth (RE_*P*_) for 12 experiments with different rainfall temporal resolutions and grid spatial resolutions. The size of the bubble represents the range of RE_*P*_. The yellow and blue colors represent that the simulated maximum inundation depth is higher and lower than the observation, respectively.

**Table 1:** Values of empirical parameters.

Number	Parameter	Value
1	Manning's roughness for impervious area	0.013
2	Manning's roughness for pervious area	0.230
3	Depression storage on impervious area (mm)	2.500
4	Depression storage on pervious area (mm)	5.000
5	Roughness of pipe	0.014
6	Maximum infiltration rate (mm·h^−1^)	104.000
7	Minimum infiltration rate (mm·h^−1^)	12.000
8	Attenuation coefficient	8.500

**Table 2:** Simulation error statistics.

	Dongcheng west road	Yonghuating	Dongzong road
NSE	0.86	0.78	0.80
RE_*P*_	11.11%	17.64%	17.50%
AE_*T*_/min	5	8	12

**Table 3:** Maximum inundation water depth at five typical waterlogging points under five temporal resolutions.

Waterlogging points	Maximum inundation water depth (cm)					
	Observation	5 min	10 min	15 min	30 min	1 h
Dongcheng west road	60	58.81	58.17	57.97	56.75	53.19
Dongzong road	25	23.65	23.61	23.34	23.21	22.19
Yonghuating	30	28.20	28.19	28.15	28.05	25.88
People's park	17	16.69	16.62	16.51	16.21	15.36
Yinshan street	22	21.17	21.11	20.90	20.84	20.12

**Table 4:** Lag time of maximum inundation depth to rainfall peak under five temporal resolutions.

Waterlogging points	Lag time (min)				
	5 min	10 min	15 min	30 min	1 h
Dongcheng west road	63	63	66	76	90
Dongzong road	80	83	83	93	116
Yonghuating	30	33	36	43	63
People's park	60	63	63	70	83
Yinshan street	63	63	66	70	86

**Table 5:** Maximum inundation depth and AE (cm) at typical waterlogging points under four spatial resolutions.

Waterlogging points	Observed value of maximum inundation depth	50 m × 50 m		100 m × 100 m		150 m × 150 m		200 m × 200 m	
		Maximum inundation depth	AE	Maximum inundation depth	AE	Maximum inundation depth	AE	Maximum inundation depth	AE
Dongcheng west road	60	61.39	−1.39	60.98	−0.98	58.81	1.19	34.13	27.26
Dongzong road	30	30.55	−0.55	29.55	0.45	28.20	2.35	23.48	7.07
Yonghuating	25	27.25	−2.50	24.00	1.00	23.65	1.35	22.82	2.18
People's park	22	22.45	−0.45	21.39	0.61	21.16	0.84	19.15	2.85
Yinshan street	17	18.20	−1.20	17.50	−0.50	16.69	0.31	15.25	1.75

## Data Availability

The rainfall records are provided by the Meteorological Bureau of Dongguan City. The data of maximum inundation depth and distribution of inundation area on May 7, 2015, were collected and released by the Water Authority of Dongguan City. The basic geographic data provided by the Urban Planning Bureau of Dongguan City included a remote-sensing image and a digital elevation model. The sewer network data was provided by the Urban Planning Bureau of Dongguan City.

## References

[1] Zheng Z., Gao J., Ma Z. (2016). Urban flooding in China: main causes and policy recommendations. *Hydrological Processes*.

[2] Wu X., Wang Z., Guo S., Liao W., Zeng Z., Chen X. (2017). Scenario-based projections of future urban inundation within a coupled hydrodynamic model framework: a case study in Dongguan city, China. *Journal of Hydrology*.

[3] Li X., Wang Y. (2022). Construction of urban flood disaster emergency management system using scenario construction technology. *Computational Intelligence and Neuroscience*.

[4] Li Z., He Y., Lu X., Zhao H., Zhou Z., Cao Y. (2021). Construction of smart city Street landscape big data-driven intelligent system based on Industry 4.0. *Computational Intelligence and Neuroscience*.

[5] Emmanuel I., Andrieu H., Leblois E., Flahaut B. (2012). Temporal and spatial variability of rainfall at the urban hydrological scale. *Journal of Hydrology*.

[6] Gires A., Tchiguirinskaia I., Schertzer D., Schellart A., Berne A., Lovejoy S. (2014). Influence of small scale rainfall variability on standard comparison tools between radar and rain gauge data. *Atmospheric Research*.

[7] Cantone J., Schmidt A. (2011). Improved understanding and prediction of the hydrologic response of highly urbanized catchments through development of the Illinois urban hydrologic model. *Water Resources Research*.

[8] Zhou Z., Smith J. A., Yang L. (2017). The complexities of urban flood response: flood frequency analyses for the Charlotte metropolitan region. *Water Resources Research*.

[9] Cao X., Lyu H., Ni G., Tian F., Ma Y., Grimmond C. S. B. (2020). Spatial scale effect of surface routing and its parameter upscaling for urban flood simulation using a grid‐based model. *Water Resources Research*.

[10] Ten Veldhuis M. C., Zhou Z., Yang L., Liu S., Smith J. (2018). The role of storm scale, position and movement in controlling urban flood response. *Hydrology and Earth System Sciences*.

[11] Schilling W. (1991). Rainfall data for urban hydrology: what do we need?. *Atmospheric Research*.

[12] Fabry F., Bellon A., Duncan M. R., Austin G. L. (1994). High resolution rainfall measurements by radar for very small basins: the sampling problem re-examined. *Journal of Hydrology*.

[13] Lyu H., Ni G., Cao X., Ma Y., Tian F. (2018). Effect of temporal resolution of rainfall on simulation of urban flood processes. *Water*.

[14] Bruni G., Reinoso R., Van de Giesen N. C., Clemens F. H. L. R., Ten Veldhuis J. A. E. (2015). On the sensitivity of urban hydrodynamic modelling to rainfall spatial and temporal resolution. *Hydrology and Earth System Sciences*.

[15] Singh V. P. (1997). Effect of spatial and temporal variability in rainfall and watershed characteristics on stream flow hydrograph. *Hydrological Processes*.

[16] Berndtsson R., Niemczynowicz J. (1988). Spatial and temporal scales in rainfall analysis — some aspects and future perspectives. *Journal of Hydrology*.

[17] Lobligeois F., Andréassian V., Perrin C., Tabary P., Loumagne C. (2013). When does higher spatial resolution rainfall information improve streamflow simulation? an evaluation using 3620 flood events. *Hydrology and Earth System Sciences Discussions*.

[18] Yang W.-Y., Li Z., Sun T., Ni G.-H. (2016). Better knowledge with more gauges? Investigation of the spatiotemporal characteristics of precipitation variations over the Greater Beijing Region. *International Journal of Climatology*.

[19] Obled C., Wendling J., Beven K. (1994). The sensitivity of hydrological models to spatial rainfall patterns: an evaluation using observed data. *Journal of Hydrology*.

[20] Cristiano E., Ten Veldhuis M. C., Van de Giesen N. (2017). Spatial and temporal variability of rainfall and their effects on hydrological response in urban areas - a review. *Hydrology and Earth System Sciences*.

[21] Aronica G., Freni G., Oliveri E. (2005). Uncertainty analysis of the influence of rainfall time resolution in the modelling of urban drainage systems. *Hydrological Processes*.

[22] Meselhe E. A., Habib E. H., Oche O. C., Gautam S. (2009). Sensitivity of conceptual and physically based hydrologic models to temporal and spatial rainfall sampling. *Journal of Hydrologic Engineering*.

[23] Gires A., Giangola-Murzyn A., Abbes J.-B., Tchiguirinskaia I., Schertzer D., Lovejoy S. (2014). Impacts of small scale rainfall variability in urban areas: a case study with 1D and 1D/2D hydrological models in a multifractal framework. *Urban Water Journal*.

[24] Ochoa-Rodriguez S., Wang L. P., Gires A. (2015). Impact of spatial and temporal resolution of rainfall inputs on urban hydrodynamic modelling outputs: a multi-catchment investigation. *Journal of Hydrology*.

[25] Yang L., Smith J. A., Baeck M. L., Zhang Y. (2016). Flash flooding in small urban watersheds: storm event hydrologic response. *Water Resources Research*.

[26] Dehotin J., Braud I. (2008). Which spatial discretization for distributed hydrological models? Proposition of a methodology and illustration for medium to large-scale catchments. *Hydrology and Earth System Sciences*.

[27] Ichiba A., Gires A., Tchiguirinskaia I., Schertzer D., Bompard P., Ten Veldhuis M.-C. (2018). Scale effect challenges in urban hydrology highlighted with a distributed hydrological model. *Hydrology and Earth System Sciences*.

[28] Amorocho J. (1961). Discussion of “predicting storm runoff on small experimental watersheds”. *Journal of the Hydraulics Division*.

[29] Minshall N. E. (1960). Predicting storm runoff on small experimental watersheds. *Journal of the Hydraulics Division*.

[30] Eddy M. (1971). *Storm Water Management Model Volume 1—Final Report*.

[31] Goldstein A., Foti R., Montalto F. (2016). Effect of spatial resolution in modeling stormwater runoff for an urban block. *Journal of Hydrologic Engineering*.

[32] Zhang W., Montgomery D. R. (1994). Digital elevation model grid size, landscape representation, and hydrologic simulations. *Water Resources Research*.

[33] Hunter N. M., Bates P. D., Neelz S. (2008). Benchmarking 2D hydraulic models for urban flooding. *Proceedings of the Institution of Civil Engineers-Water Management*.

[34] Russo B., Sunyer D., Velasco M., Djordjević S. (2015). Analysis of extreme flooding events through a calibrated 1D/2D coupled model: the case of Barcelona (Spain). *Journal of Hydroinformatics*.

[35] Yu W., Ma J., Yin Y., Yu H., Wu B., Mu J. (2022). 2D Hydrodynamic model based on adaptive grid. *China Flood & Drought Management*.

